# Global Analysis and Optimal Control Model of COVID-19

**DOI:** 10.1155/2022/9491847

**Published:** 2022-01-27

**Authors:** Sacrifice Nana-Kyere, Francis Agyei Boateng, Paddy Jonathan, Anthony Donkor, Glory Kofi Hoggar, Banon Desmond Titus, Daniel Kwarteng, Isaac Kwasi Adu

**Affiliations:** ^1^Deparment of Mathematics and Information Technology, Valley View University, Ghana; ^2^Department of Agriculture Economics, Agribusiness and Extension, University of Energy and Natural Resources, Ghana; ^3^Department of Computer Science and Mathematics, Sunyani Technical University, Ghana; ^4^Budget Department, Wenchi Municipal Assembly, Ghana; ^5^Department of Mathematics, Kibi College of Education, Ghana; ^6^Mathematical Science Department, Kumasi Technical University, Ghana

## Abstract

COVID-19 remains the concern of the globe as governments struggle to defeat the pandemic. Understanding the dynamics of the epidemic is as important as detecting and treatment of infected individuals. Mathematical models play a crucial role in exploring the dynamics of the outbreak by deducing strategies paramount for curtailing the disease. The research extensively studies the SEQIAHR compartmental model of COVID-19 to provide insight into the dynamics of the disease by underlying tailored strategies designed to minimize the pandemic. We first studied the noncontrol model's dynamic behaviour by calculating the reproduction number and examining the two nonnegative equilibria' existence. The model utilizes the Castillo-Chavez method and Lyapunov function to investigate the global stability of the disease at the disease-free and endemic equilibrium. Sensitivity analysis was carried on to determine the impact of some parameters on *R*_0_. We further examined the COVID model to determine the type of bifurcation that it exhibits. To help contain the spread of the disease, we formulated a new SEQIAHR compartmental optimal control model with time-dependent controls: personal protection and vaccination of the susceptible individuals. We solved it by utilizing Pontryagin's maximum principle after studying the dynamical behaviour of the noncontrol model. We solved the model numerically by considering different simulation controls' pairing and examined their effectiveness.

## 1. Introduction

The unusual, life-threatening pneumonia condition affecting humanity remains the globe's concern as governments struggle to defeat the pandemic. COVID-19, one of the most media campaigned viral diseases, emerged from Wuhan's city in China in the last quarter of 2019. The epidemic has transcended the nations' regions, and all sectors of the global economy have felt its adverse effects [1]. The epidemic has been the source of setbacks in businesses, disruption in academic calendars, and closure of production companies and public services [2]. The campaign against the disease has intensified due to the number of case counts and deaths recorded each day globally. The primary mode of transmissibility of the disease is airborne. Thus, individuals become infected by contact with the contaminated sneezes and droplets of the virus [3]. The documented number of COVID-19-related deaths and cases in the first quarter of the year 2020 caused governments to respond accordingly by promoting and observing self-protective protocols and restrictions directed by the World Health Organization. However, the protocols and restrictions were gradually eased when evidence of the disease waning was confirmed by governments [4]. Notably, the vast majority of the European countries are currently battling with the second wave of COVID-19 outbreaks after successfully minimizing COVID-19 disease in the early months of the year 2020 [5]. The second wave has caused the European countries' governments to respond to the second spike by introducing new measures that may help manage the disease and prevent the further spread of the outbreak. These measures range from strict new restrictions, such as minilockdown and compulsory mask wearing, to relaxed regulations, allowing the opening of bars and pubs with a set time for closure. These recommended restrictions vary from country to country regarding the number of cases and infection rates [6].

Since the detection of the virus in Wuhan, variants of COVID-19 mathematical models have been considered that have helped shape the pandemic, with inked preventive measures which could be adopted to flatten the curve, estimating the final epidemic size and prevent further infection (see [7–23]).

Mathematical modelling of infectious diseases has been an experimenting station where the vast knowledge of epidemic outbreaks, transmission dynamics, intervention, and alternative courses of action for controlling diseases are discovered. Integrating mathematical computation into the modelling of infectious diseases has evolved in an unparalleled achievement regarding intervention strategies and has been the spine of all explorations on infectious diseases [24].

In their paper, Hellewell et al. [25] assessed the effectiveness of a stochastic transmission model to control the new SARS-CoV-2 disease by utilizing the preventive measures of isolation and contact tracing. Qianying et al. [26], in their work, constructed SEIRNDC compartmental model of coronavirus-2 in Wuhan that examines the government's responses towards the disease and the reaction from the people. The authors in [27] considered an eight compartmental nonlinear differential equation model of COVID-19 that uses time-dependent diagnosis and contact rates to refit their existing SEIR compartmental model [28] to a newly available data for better estimation of the basic reproduction number. In a related paper, Kang et al. [29] examined the COVID-19 epidemic dynamics in China. The authors applied Moran's I spatial statistics in a test to ascertain the possibility of the disease's spatial association. In [30], in their paper, the author adapted the growth model to study the spread pattern of MERS, COVID-19, and SARS by using the inhibition and growth rates to establish the model's propagation. Benvenuto et al. [31] predicted the spread and trend of COVID-19 disease by using the ARIMA model. In a paper related to the current studies, Li et al. [32] investigated the COVID-19 transmission process using the official modelling data. The study examines the error between the model and the official data. In [7], in their work, the authors calibrated a COVID-19 epidemic model to deduce various characteristics such as age-dependent attack rates, length of incubation, generation periods, reproductive number, and growth rate of cumulative incidence. In [10], in their research, the authors analyzed the spread pattern of the COVID-19 outbreak by using a time series model. The authors in [33] considered variants of the SIR model with a parameter that factors into account the effects of social distancing. Fu et al. [34] applied Boltzmann-function-based regression analyses to estimate the number of SARS-CoV-2 confirmed cases in China. Shi et al. [35] considered a SEIR COVID-19 propagation model that assessed the variation in the length of the incubation period, weakness of the transmission ability of the incubation period, and the intervention of the government to detect and isolate the infected. In [36], the authors studied and predicted the pattern of the COVID-19 epidemic and estimated the various parameters involved in the model's analyses. Liu et al. [37] considered a new QSEIR COVID-19 epidemic model that studied the effect of quarantine measures imposed in Mainland China during the peak of the outbreak. In [38], in their paper, a stochastic COVID-19 transmission model is examined that analyzed the intervention measures employed in Mainland China. Kissler et al. [39] applied a mathematical model to prove that the United States' critical care capacity will not be sufficient to be maintained with a one-time intervention strategy. In [40], the authors fitted a coronavirus-2 age-structured model to data from six countries affected by the pandemic to determine the age gradient in observed cases. In [41], the authors studied a SEIR compartmental model of COVID-19, with modifications to account for the spreading of the epidemic in the latent stage and the effects of varying containment's proportions. Acuna et al. [42] considered mathematical models which examine the issues related to the spread of SARS-CoV-2 in Mexico and explore the effect of behaviour changes needed to wane the infection. Rong et al. [43] studied a new dynamical model of SS_q_EI_1_I_2_HRV for SARS-CoV-2 to assess the effect of delay in detecting an infected person. In a related article, Giordano et al. [44], considered a nonlinear ordinary differential equation model of SIDARTHE compartments that predicts the propagation of COV-19 epidemic in Italy and helps to diffuse the misperceptions of epidemic spread and case fatality rate. In [45], the authors in their work explored the impact of community mask wearing on COVID-19 transmission dynamics in the United States by formulating a new mathematical model for the assessment.

Optimal control models have engineered tailored strategies that have been paramount for minimizing and prevention of infections [46–56].

Asamoah et al. [57] applied an optimal control theory to nonlinear ordinary differential equations of SEAIRV compartmental model of coronavirus transmission that analyzed the cost-effective strategy of all the proposed methods. In the paper by [58], the authors constructed and researched a compartmental SIRU model that brings further insight into the propagation of the COVID-19 disease. The SIRU compartmental model is then converted to an optimal control problem, and the numerical solutions are presented. The authors in [59] formulated a mathematical model for coronavirus-2 disease to estimate the model parameters by fitting it to actual data. The authors further performed optimal control analysis on the modified model. In [30], the author constructed a mathematical model that is segregated into compartments of SEIRV for the coronavirus-2 epidemic and converted it to an optimal control problem by characterizing several control strategies by applying the maximum principle. Sasmita et al. [60] considered SEI_1_I_2_RS nonlinear compartmental model of coronavirus-2 infection to predict the disease's peak in Indonesia. The authors considered five time-dependent controls in constructing the optimal control model to deduce strategies critical for policymakers to curb the pandemic. The authors in [61] applied an optimal control analysis to a mathematical model of SARS-CoV-19 to help deduce many possible strategies for the control of the disease. In [62], the authors developed an ordinary differential equation model of SEIRW compartments that describes the COVID-19 disease's dynamics. The authors made a SEIRW compartmental model modification to convert the dynamical model into a new SEIRW control model to assess the chosen strategies thoroughly.

This research article presents a SEQIAHR compartmental model of COVID-19 to provide insight into the disease's dynamics by utilizing tailored strategies to minimize the pandemic. The study is motivated by the available COVID-19 works and formulating a new SEQIAHR compartmental optimal control model that would add to the existing knowledge and help improve public health decision-making by providing scientific strategies to prevent the disease.

The remaining work is organized as follows: Section 2 formulates a deterministic SEQIAHR compartmental COVID-19 model.  Section 3 studies the global stability of the model, sensitivity and bifurcation analysis. A new SEQIAHR compartmental optimal control model is constructed and analyzed in Section 4 with time-dependent control functions of personal protection and treatment of asymptomatic infected individuals. Finally, Section 5 discusses the simulated results of the models by using an iterative method of Runge-Kutta 4th-order method and Matlab.

## 2. The Model Formulation

This section formulates a compartmental SEQIAHR transmission model for COVID-19 disease to understand the dynamical behaviour of the disease and the strategy needed in curtailing it. Here, we modify the baseline model of [45] which is segregated into compartments of: susceptible *S*(*t*), exposed *E*(*t*), symptomatic infectious *I*(*t*), asymptomatic infectious *A*(*t*), hospitalized *H*(*t*), recovered *R*(*t*), and cumulative deaths *D*(*t*), by considering recruitment into the population, *Λ* and natural death rate *μ*, and ignoring the cumulative death compartment. Additionally, we assume that COVID-19 has a high level of transmission, and therefore, the main way of preventing the spread of the disease is to adopt a quarantine approach of the exposed individuals. This is considered in the formulation of the model by first modifying the original model system (1) of [45], with the inclusion of quarantine compartment, by assuming that the exposed individuals are quarantined at rate *τ*. Further, the model assumes that the quarantine individuals are hospitalized at a rate of *τ*_1_. Also, we assume that the quarantined individuals may die naturally. We assumed a time-dependent population for the modified model. With these assumptions, the modified model equations are given as follows:

(1) $$\begin{array}{c} \left\{\begin{array}{c} \frac{d}{dt}S=\Lambda -\frac{\beta SI}{N}-\frac{\beta S\eta A}{N}-\mu S,\\ \frac{d}{dt}E=\frac{\beta SI}{N}+\frac{\beta S\eta A}{N}-\sigma E-\tau E-\mu E,\\ \frac{d}{dt}Q=\tau E-\left(\tau_{1}+\mu \right)Q,\\ \frac{d}{dt}I=\alpha \sigma E-\phi I-\gamma_{I}I-\mu I,\\ \frac{d}{dt}A=\left(1-\alpha \right)\sigma E-\gamma_{A}A-\mu A,\\ \frac{d}{dt}H=\phi I+\tau_{1}Q-\delta H-\gamma_{H}H-\mu H,\\ \frac{d}{dt}R=\gamma_{I}I+\gamma_{A}A+\gamma_{H}H-\mu R, \end{array}\right. \end{array}$$

with *S* ≥ 0, *E* ≥ 0, *Q* ≥ 0, *I* ≥ 0, *A* ≥ 0, *H* ≥ 0, and *R* ≥ 0.

### 2.1. Analysis of Model: Positivity and Boundedness

**Theorem 1 .**

The set {*S*(*t*), *E*(*t*), *Q*(*t*), *I*(*t*), *A*(*t*), *H*(*t*), *R*(*t*)} being the solution of the state Equation (1) with nonnegative parameters is positive with initial conditions given by the following:

(2) $$\begin{array}{c} \left\{S\left(0\right)\geq 0,E\left(0\right)\geq 0,Q\left(0\right)\geq 0,I\left(0\right)\geq 0,A\left(0\right)\geq 0,H\left(0\right)\geq 0,R\left(0\right)\geq 0\right\}. \end{array}$$

**Proof**

With the method illustrated by [57], theorem one can be proofed by adopting the same approach as underlaid below.

We redefine *W* = (*S*, *E*, *Q*, *I*, *A*, *H*, *R*)^*T*^, *U*_0_ = (*β*/*N*)*I*, and *U*_1_ = (*βη*/*N*)*A*, with *T* denoting the transposition. Hence, COVID-19 model Equation (1) in matrix form is represented as follows:

(3) $$\begin{array}{c} \frac{dW}{dt}=PW+B, \end{array}$$

where

(4) $$\begin{array}{c} P=\left(\begin{array}{ccccccc} -\left(U_{0}+U_{1}+\mu \right) & 0 & 0 & 0 & 0 & 0 & 0\\ \left(U_{0}+U_{1}\right) & -\left(\sigma +\tau +\mu \right) & 0 & 0 & 0 & 0 & 0\\ 0 & \tau & -\left(\tau_{1}+\mu \right) & 0 & 0 & 0 & 0\\ 0 & \alpha \sigma & 0 & -\left(\phi +\gamma_{I}+\mu \right) & 0 & 0 & 0\\ 0 & \left(1-\alpha \right)\sigma & 0 & 0 & -\left(\gamma_{A}+\mu \right) & 0 & 0\\ 0 & 0 & \tau_{1} & \phi & 0 & -\left(\delta +\gamma_{H}+\mu \right) & 0\\ 0 & 0 & 0 & \gamma_{I} & \gamma_{A} & \gamma_{H} & -\mu \end{array}\right),\\ B=\left(\begin{array}{c} \Lambda \\ 0\\ 0\\ 0\\ 0\\ 0\\ 0 \end{array}\right). \end{array}$$

In model Equation (1), rewriting the third equation into a first-order nonhomogenous differential equation gives

(5) $$\begin{array}{c} \frac{dQ}{dt}+\left(\tau_{1}+\mu \right)Q=\tau E. \end{array}$$

Now, from (5), adopting the method of integrating factor and applying it provides

(6) $$\begin{array}{c} Q\left(t\right)=e^{-\left(\tau_{1}+\mu \right)t}\left[Q\left(0\right)+\tau \int_{0}^{t}E\left(s\right)e^{-\left(\tau_{1}+\mu \right)s}.ds\right]. \end{array}$$

Similarly, mimicking the same approach, the fourth equation of model (1) gives

(7) $$\begin{array}{c} I\left(t\right)=e^{-\left(\phi +\gamma_{I}+\mu \right)t}\left[I\left(0\right)+\alpha \sigma \int_{0}^{t}E\left(s\right)e^{-\left(\phi +\gamma_{I}+\mu \right)s}.ds\right]. \end{array}$$

Now, as can be determined in the work of [57], it follows that by intuition, (*d*/*dt*)*Q* ≥ 0, at *t* = 0, and (*d*/*dt*)*I* ≥ 0, at *t* = 0, for *E*(0) = 0. Hence, following the same steps, the same can be generalized for *S*(*t*), *E*(*t*), *A*(*t*), *H*(*t*), and *R*(*t*), which ensures that the state variables stays positive in the entire time of the study. In addition, by inspection, it could be verified that the off-diagoanl entries of *P* are nonnegative and *B* ≥ 0, which confirms the property Metzler matrix [57]. Hence, the state model Equation (1) is positively invariant in *R*_+_^7^.

**Theorem 2 .**

The nonlinear equation model (1) has solutions bounded within the invariant region, *φ* ∈ *R*^7^ given as

(8) $$\begin{array}{c} \varphi =\left\{\left(S,E,Q,I,A,H,R\right)\in R_{+}^{7},S+E+Q+I+A+H+R\leq \Lambda -\delta H-\mu N\right\}. \end{array}$$

**Proof**

Here, we denote *N*(*t*) = *S* + *E* + *Q* + *I* + *A* + *H* + *R*. Then, the simplified nonlinear differential equation of (1) is given as

(9) $$\begin{array}{c} \frac{d}{dt}N\left(t\right)=\Lambda -\delta H-\mu N. \end{array}$$

Then, from Equation (9), setting *Z* to be a solution of (9) gives a unique initial value problem

(10) $$\begin{array}{c} \left\{\begin{array}{cc} \frac{d}{dt}Z_{1}\left(t\right)=\Lambda -\mu Z_{1}\left(t\right) & \text{for }t\geq 0,\\ Z_{1}\left(0\right)=N\left(0\right). \end{array}\right. \end{array}$$

Solving Equation (54) produces

(11) $$\begin{array}{c} Z_{1}\left(t\right)=N\left(0\right)e^{-\mu t}+\frac{\Lambda }{\mu }\left(1-e^{\left(-\mu t\right)}\right). \end{array}$$

Hence, from the comparison theorem [63], it can be seen that

(12) $$\begin{array}{c} N\left(t\right)=N\left(0\right)e^{-\mu t}+\frac{\Lambda }{\mu }\left(1-e^{\left(-\mu t\right)}\right). \end{array}$$

Therefore, from (12), it follows that the possible solution set of the state variables *S*, *E*, *Q*, *I*, *A*, *H*, *R* is bounded and the state model Equation (1) is positively in variant in *R*_+_^7^, implying that any trajectory with initial condition in *R*_+_^7^ will remain in *φ*. This guarantees that model (1) is mathematically and epidemiologically feasible and well posed.

### 2.2. Disease-Free Equilibrium and Reproduction Ratio

The basic reproduction number threshold parameter is key in determining whether an invading infection from an infected individual will have the potency to be endemic or die out in a naive population. It is defined as a new infection from an infected individual who enters into a naive susceptible population. When *R* = 0, *H* = 0, *A* = 0, *I* = 0, *Q* = 0, and *E* = 0, then the COVID-19 model (1) has a disease-free equilibrium (DFE), determined by equating the right-hand side of the equations in model (1) to zero and solve for the state variables. Hence,

(13) $$\begin{array}{c} E_{0}=\left(S_{0},E_{0},Q_{0},I_{0},A_{0},H_{0},R_{0}\right)=\left(\frac{\Lambda }{\mu },0,0,0,0,0,0\right). \end{array}$$

The basic reproduction number of the model system (1) at *E*_0_ = (*S*_0_, *E*_0_, *Q*_0_, *I*_0_, *A*_0_, *H*_0_, *R*_0_) is derived from the method studied in [64] by Diekmann et al. Based on [64], we derive matrices *F* and *V* as follows:

(14) $$\begin{array}{c} F_{J}=\left(\begin{array}{cccc} 0 & 0 & \beta & \beta \eta \\ 0 & 0 & 0 & 0\\ 0 & 0 & 0 & 0\\ 0 & 0 & 0 & 0 \end{array}\right),\\ V=\left(\begin{array}{cccc} \left(\sigma +\tau +\mu \right) & 0 & 0 & 0\\ -\tau & \left(\tau_{1}+\mu \right) & 0 & 0\\ -\alpha \sigma & 0 & \left(\phi +\gamma_{I}+\mu \right) & 0\\ -\left(1-\alpha \right)\sigma & 0 & 0 & \left(\gamma_{A}+\mu \right) \end{array}\right). \end{array}$$

Hence, the basic reproduction number for the COVID-19 model (1) is obtained by the spectral radius of *ρ*(*FV*^−^1) as follows:

(15) $$\begin{array}{c} R_{0}=\frac{\alpha \sigma \beta }{\left(\sigma +\tau +\mu \right)\left(\phi +\gamma_{I}+\mu \right)}+\frac{\left(1-\alpha \right)\eta \sigma \beta }{\left(\sigma +\tau +\mu \right)\left(\gamma_{A}+\mu \right)}. \end{array}$$

### 2.3. Existence of Endemic Equilibrium

When *R* ≠ 0, *H* ≠ 0, *A* ≠ 0, *I* ≠ 0, *Q* ≠ 0, *E* ≠ 0, and *S* ≠ 0, then it follows that the endemic equilibrium exists. This unique equilibrium point for the COVID-19 model system (1) given by *E*_1_^∗^ = (*S*^∗^, *E*^∗^, *Q*^∗^, *I*^∗^, *A*^∗^, *H*^∗^, *R*^∗^) is determined as follows:

(16) $$\begin{array}{c} \left\{\begin{array}{c} S^{*}=\frac{1}{R_{0}},\\ E^{*}=\frac{\mu \left(NR_{0}-1\right)\left(\phi +\gamma_{I}+\mu \right)\left(\gamma_{A}+\mu \right)N}{\beta \sigma \left(\alpha \left(\gamma_{A}+\mu \right)+\eta \left(1-\alpha \right)\left(\phi +\gamma_{I}+\mu \right)\right)},\\ Q^{*}=\frac{\mu \tau_{1}\left(NR_{0}-1\right)\left(\phi +\gamma_{I}+\mu \right)\left(\gamma_{A}+\mu \right)N}{\beta \sigma \left(\xi +\mu \right)\left(\alpha \left(\gamma_{A}+\mu \right)+\eta \left(1-\alpha \right)\left(\phi +\gamma_{I}+\mu \right)\right)},\\ I^{*}=\frac{\alpha \sigma \mu \left(NR_{0}-1\right)\left(\gamma_{A}+\mu \right)N}{\beta \sigma \left(\alpha \left(\gamma_{A}+\mu \right)+\eta \left(1-\alpha \right)\left(\phi +\gamma_{I}+\mu \right)\right)},\\ A^{*}=\frac{\left(1-\alpha \right)\sigma \mu \left(NR_{0}-1\right)\left(\phi +\gamma_{I}+\mu \right)N}{\beta \sigma \left(\alpha \left(\gamma_{A}+\mu \right)+\eta \left(1-\alpha \right)\left(\phi +\gamma_{I}+\mu \right)\right)},\\ H^{*}=\frac{\left(NR_{0}-1\right)\left(\gamma_{A}+\mu \right)\mu N\left[\phi \alpha \sigma +\tau_{1}\left(\phi +\gamma_{I}+\mu \right)\right]}{\beta \sigma \left(\alpha \left(\gamma_{A}+\mu \right)+\eta \left(1-\alpha \right)\left(\phi +\gamma_{I}+\mu \right)\right)},\\ R^{*}=\frac{\sigma \mu \left(NR_{0}-1\right)\left(\alpha \gamma_{I}\left(\gamma_{A}+\mu \right)+\gamma_{A}\left(1-\alpha \right)\left(\phi +\gamma_{I}+\mu \right)+\alpha \phi \eta \gamma_{H}\left(\gamma_{A}+\mu \right)\right)}{\beta \sigma \left(\alpha \left(\gamma_{A}+\mu \right)+\eta \left(1-\alpha \right)\left(\phi +\gamma_{I}+\mu \right)\right)}. \end{array}\right. \end{array}$$

## 3. Disease-Free Equilibrium (DFE) and Its Stability

In this section, the global stability analysis of the COVID-19 model (1) at the disease-free equilibrium is studied. The Castillo-Chavez method [65] would be used to prove that model (1) is globally asymptotically stable at the disease-free equilibrium. Thus, it follows that in considering the method of Castillo-Chavez, the COVID-19 model (1) can be transformed as follows:

(17) $$\begin{array}{c} \frac{dp_{1}}{dt}=y_{1}\left(p_{1},p_{2}\right),\\ \frac{dp_{2}}{dt}=y_{2}\left(p_{1},p_{2}\right),y_{2}\left(p_{1},0\right)=0, \end{array}$$

where *p*_1_ denotes the uninfected population; thus, *p*_1_ = (*S*, *R*), and *p*_2_ represents the infected, with, *p*_2_ = (*E*, *Q*, *I*, *A*, *H*). The disease-free equilibrium point of (1) is given by *U* = (*p*_1_^0^, 0).

The point (*y*_1_^0^, 0) is a globally stable asymptotically stable equilibrium for the model (1) provided *R*_0_ < 1, and the below criteria are satisfied.

*D1*. Given *dp*_1_/*dt* = *y*_1_(*p*_1_, 0), (*p*_1_^0^) is globally asymptotically stable.

*D2*. $y\left(p_{1},p_{2}\right)=Zp_{2}-{\hat{y}}_{2}\left(p_{1},p_{2}\right)$, where ${\hat{y}}_{2}\left(p_{1},p_{2}\right)\geq 0$ for (*p*_1_, *p*_2_) ∈ *ζ*_*u*._

What happens next is if the model Equation (1) meets the above conditions; then, the following theorem holds.

**Theorem 3 .**

The point *U* = (*p*_1_^0^, 0) is globally asymptotically stable equilibrium given that *R*_0_ < 1 and the conditions D1 and D2 are satisfied.

**Proof**

Concerning the model Equation (1), we derive *y*_1_(*p*_1_, *p*_2_) and *y*_2_(*p*_1_, *p*_2_) as

(18) $$\begin{array}{c} y_{1}\left(p_{1},p_{2}\right)=\left(\begin{array}{c} \Lambda -\frac{\beta SI}{N}-\frac{\beta S\eta A}{N}-\mu S\\ \gamma_{I}I+\gamma_{A}A+\gamma_{H}H-\mu R \end{array}\right),\\ y_{2}\left(p_{1},p_{2}\right)=\left(\begin{array}{c} \frac{\beta SI}{N}+\frac{\beta S\eta A}{N}-\sigma E-\tau E-\mu E\\ \tau E-\left(\tau_{1}+\mu \right)Q\\ \alpha \sigma E-\phi I-\gamma_{I}I-\mu I\\ \left(1-\alpha \right)\sigma E-\gamma_{A}A-\mu A\\ \phi I+\tau_{1}Q-\delta H-\gamma_{H}H-\mu H \end{array}\right). \end{array}$$

It follows that with *S* = *S*_0_, *I* = *I*_0_, *A* = *A*_0_, *H* = *H*_0_, and *R* = *R*_0_, then *y*_1_(*p*_1_, 0) becomes

(19) $$\begin{array}{c} y_{1}\left(p_{1},p_{2}\right)=\left(\begin{array}{c} \Lambda -\frac{\beta S_{0}I_{0}}{N}-\frac{\beta S_{0}\eta A_{0}}{N}-\mu S_{0}\\ \gamma_{I}I_{0}+\gamma_{A}A_{0}+\gamma_{H}H_{0}-\mu R_{0} \end{array}\right). \end{array}$$

What follows next is that from (19), we notice that as *t*⟶∞, *p*_1_ = *p*_1_^0^. Hence, *p*_1_ = *p*_1_^0^ is globally asymptotically stable, which verifies the first condition.

Now, in determining whether condition two would be satisfied, we utilize $Y\left(p_{1},p_{2}\right)=Zp_{2}-{\hat{y}}_{2}\left(p_{1},p_{2}\right)$. And we get

(20) $$\begin{array}{c} A=\left(\begin{array}{ccccc} -a_{11} & 0 & \frac{\beta }{N}S_{0} & \frac{\beta \eta }{N}S_{0} & 0\\ \tau & -a_{22} & 0 & 0 & 0\\ \alpha \sigma & 0 & -a_{33} & 0 & 0\\ \left(1-\alpha \right)\sigma & 0 & 0 & -a_{44} & 0\\ 0 & \tau_{1} & \phi & 0 & -a_{55} \end{array}\right)\left(\begin{array}{c} E\\ Q\\ I\\ A\\ H \end{array}\right)-\left(\begin{array}{c} {\hat{y}}_{2}\left(p_{1},p_{2}\right)\\ 0\\ 0\\ 0\\ 0 \end{array}\right), \end{array}$$

where $𝒜=Dy_{2}-{\hat{\text{W}}}_{2}\left(y_{1},y_{2}\right)$, *a*_11_ = (*σ* + *τ* + *μ*), *a*_22_ = (*τ*_1_ + *μ*), *a*_33_ = (*ϕ* + *γ*_*I*_ + *μ*), *a*_44_ = (*γ*_*A*_ + *μ*), *a*_55_ = (*δ* + *γ*_*H*_ + *μ*), and matrix *D* given by

(21) $$\begin{array}{c} Z=\left(\begin{array}{ccccc} -a_{11} & 0 & \frac{\beta }{N}S_{0} & \frac{\beta \eta }{N}S_{0} & 0\\ \tau & -a_{22} & 0 & 0 & 0\\ \alpha \sigma & 0 & -a_{33} & 0 & 0\\ \left(1-\alpha \right)\sigma & 0 & 0 & -a_{44} & 0\\ 0 & \tau_{1} & \phi & 0 & -a_{55} \end{array}\right), \end{array}$$

with

(22) $$\begin{array}{c} J=\left(\begin{array}{cc} \beta \left(S_{0}-S\right)\frac{I}{N} & \beta \eta \left(S_{0}-S\right)\frac{I}{N}\\ 0 & 0\\ 0 & 0\\ 0 & 0\\ 0 & 0 \end{array}\right), \end{array}$$

where $𝒥={\hat{y}}_{2}\left(p_{1},p_{2}\right)$. It can be ascertained from model Equation (1) that the total population is bounded by *S*_0_. Therefore, it follows that (*βI*/*N*)*S* ≤ (*βI*/*N*)*S*_0_, and *η*(*βI*/*N*)*S* ≤ *η*(*βI*/*N*)*S*_0_ which implies ${\hat{y}}_{2}\left(p_{1},p_{2}\right)$ is positive definite. Further, matrix *Z* is evidently an M-matrix, with the off-diagonal entries positive. Hence, condition two is satisfied which proves the global asymptotic stability of *U*.

### 3.1. Endemic Equilibrium (EE) and Its Stability

This subsection presents the global stability analysis of the COVID-19 model (1) at the endemic equilibrium by applying a Lyapunov function theory [66] for the global stability analysis. The results are given as follows:

**Theorem 4 .**

The unique endemic equilibrium *E*_1_^∗^ for the COVID-19 model (1) is globally asymptotically stable in *R*+^7^ whenever *R*_0_ > 1.

**Proof**

The Lyapunov function *L* = *m*_1_*S* + *m*_2_*E* + *m*_3_*Q* + *m*_4_*I* + *m*_5_*A* + *m*_6_*H* + *m*_7_*R*, where *m*_*i*_ for *i* = 1, 2, 3 ⋯ .7 are constants to be chosen in the course of the proof are defined.

The derivative of *L* along the solution of (1) is given by

(23) $$\begin{array}{c} \frac{dL}{dt}=m_{1}\frac{dS}{dt}+m_{2}\frac{dE}{dt}+m_{3}\frac{dq}{dt}+m_{4}\frac{dI}{dt}+m_{5}\frac{dA}{dt}+m_{6}\frac{dH}{dt}+m_{7}\frac{dR}{dt},\\ \frac{dL}{dt}=m_{1}\left(\Lambda -\frac{\beta \left(I+\eta A\right)S}{N}-\mu S\right)+m_{2}\left(\frac{\beta \left(I+\eta A\right)S}{N}-\sigma E-\tau E-\mu E\right)+m_{3}\left(\tau E-\left(\tau_{1}+\mu \right)Q\right)+m_{4}\left(\alpha \sigma E-\phi I-\gamma_{I}I-\mu I\right)+m_{5}\left(\left(1-\alpha \right)\sigma E-\gamma_{A}A-\mu A\right)+m_{6}\left(\phi I+\tau_{1}Q-\delta H-\gamma_{H}H-\mu H\right)+m_{7}\left(\gamma_{I}I+\gamma_{A}A+\gamma_{H}H-\mu R\right),\\ \frac{dL}{dt}=m_{1}\left(\Lambda -\mu S\right)+\left(m_{2}-m_{1}\right)\frac{\beta \left(I+\eta A\right)S}{N}+\left(m_{5}-m_{2}\right)\sigma E+\left(m_{3}-m_{2}\right)\tau E-m_{2}\mu E+\left(m_{6}-m_{3}\right)\tau_{1}Q-m_{3}\mu Q+\left(m_{4}-m_{5}\right)\alpha \sigma E+\left(m_{6}-m_{4}\right)\phi I+\left(m_{7}-m_{4}\right)\gamma_{I}I-m_{4}\mu I+\left(m_{7}-m_{5}\right)\gamma_{A}A-m_{5}\mu A-m_{6}\delta H-m_{6}\mu H+\left(m_{7}-m_{6}\right)\gamma_{H}H-m_{7}\mu R. \end{array}$$

Choosing *m*_1_, *m*_2_, *m*_3_, *m*_4_, *m*_5_, *m*_6_, and *m*_7_ such that *m*_1_ = *m*_2_ = *m*_3_ = *m*_4_ = *m*_5_ = *m*_6_ = *m*_7_ and *Λ* − *μS* = 0 gives

(24) $$\begin{array}{c} -m_{2}\mu E-m_{3}\mu Q-m_{4}\mu I-m_{5}\mu A-m_{6}\delta H-m_{6}\mu H-m_{7}\mu R. \end{array}$$

It follows that *L* is positive definite, and *dL*/*dt* is negative definite. Therefore, the function *L* is a Lyapunov function for model system (1), and by Lyapunov asymptotic stability theorem [67], the endemic equilibrium *E*_1_^∗^ is globally asymptotically stable.

### 3.2. Sensitivity Analysis

Sensitivity analysis is one of the essential subjects that has been explored by many researchers and is of great importance to epidemiological modelling. Sensitivity analysis study assists us in ascertaining parameters that impact the *R*_0_ and allows epidemiologists to improve the design of the control strategies. The results from sensitivity index computation indicate the effect of involving parameters that contribute to the spreading of the epidemic and inform us of the relative change of *R*_*o*_ and other parameters.

**Definition 1 .**

For a given parameter *α*, the normalized forward sensitivity index of *R*_0_ is computed using the formula discussed in [18, 68], as

(25) $$\begin{array}{c} \varsigma_{\alpha }^{R_{0}}=\frac{\partial R_{0}}{\partial \alpha }\frac{\alpha }{R_{0}}. \end{array}$$

Applying this formula for the parameters *β* and *α* gives

(26) $$\begin{array}{c} \frac{\partial R_{0}}{\partial \beta }\frac{\beta }{R_{0}}=\frac{\alpha \sigma \left(\gamma_{A}+\mu \right)+\left(1-\alpha \right)\eta \sigma \left(\phi +\gamma_{I}+\mu \right)}{\left(\sigma +\tau +\mu \right)\left(\phi +\gamma_{I}+\mu \right)\left(\gamma_{A}+\mu \right)}.\beta \frac{\left(\sigma +\tau +\mu \right)\left(\phi +\gamma_{I}+\mu \right)\left(\gamma_{A}+\mu \right)}{\alpha \sigma \beta \left(\gamma_{A}+\mu \right)+\left(1-\alpha \right)\eta \sigma \beta \left(\phi +\gamma_{I}+\mu \right)}=1,\\ \frac{\partial R_{0}}{\partial \alpha }\frac{\alpha }{R_{0}}=\frac{\left(1-\alpha \right)\sigma \beta }{\left(\sigma +\tau +\mu \right)\left(\gamma_{A}+\mu \right)}.\eta \frac{\left(\sigma +\tau +\mu \right)\left(\phi +\gamma_{I}+\mu \right)\left(\gamma_{A}+\mu \right)}{\alpha \sigma \beta \left(\gamma_{A}+\mu \right)+\left(1-\alpha \right)\eta \sigma \beta \left(\phi +\gamma_{I}+\mu \right)}=\frac{\left(1-\alpha \right)\sigma \eta }{\alpha \sigma \beta \left(\gamma_{A}+\mu \right)+\left(1-\alpha \right)\eta \sigma \beta \left(\phi +\gamma_{I}+\mu \right)}. \end{array}$$

Mimicking the above method for the remaining parameters and evaluating the results with the parameter values of Table 1 provide the sensitivity indices of *R*_0_ parameters presented in Table 2.

As noted from Table 2, *β*, *η*, and *α* are the parameters with positive indices contributing to the spreading of the epidemic. The positive parameters contribute to the spreading of the outbreak since they increase the *R*_0_. On the other hand, the parameters with a negative index contribute to controlling the disease since they have reduced the *R*_0_. Further, as noted, the parameter *β* has a sensitivity index of +1, which implies increasing or decreasing *β* by a specific percentage increases or reduces *R*_0_ by the same percentage.

### 3.3. Bifurcation Analysis

In an attempt to ascertain whether model system (1) exhibits backward bifurcation or not, we analyze model system (1) with the theory of centre manifold as credited to Castillo-Chavez and Song in ([69] see Theorem 6).

Hence, we use the approach of ([69, 70]) to determine the criteria on which the parameter values of model system (1) cause a backward or forward bifurcation to occur. We consider the system below:

(27) $$\begin{array}{c} \frac{d}{dt}x=f\left(x,\in_{1}\right), \end{array}$$

where *f* is continously differentiable at least twice in *x* and ∈_1_ is the bifurcation parameters.

Equations *a* and *b* are denoted by as follows:

(28) $$\begin{array}{c} a=\overset{n}{\underset{k,i,j=1}{\sum }}\frac{v_{k}w_{i}w_{j}\partial^{2}f_{k}\left(0,0\right)}{\partial x_{i}\partial x_{j}} \end{array}$$

and

(29) $$\begin{array}{c} b=\overset{n}{\underset{k,i,j=1}{\sum }}\frac{v_{k}w_{i}\partial^{2}f_{k}\left(0,0\right)}{\partial x_{i}\partial \in_{1}} \end{array}$$

are the determinants of the existence of bifurcation in model system (1). Thus, when *a* > 0 and *b* > 0, then backward bifurcation exists and occurs at ∈_1_ = 0. When *a* < 0 and *b* > 0, forward bifurcation exists and occurs at ∈_1_ = 0. Now, considering *β* as a bifurcation parameter, then *R*_0_ be equivalent to

(30) $$\begin{array}{c} \beta =\beta^{*}=\frac{\left(\sigma +\tau +\mu \right)\left(\phi +\gamma_{I}+\mu \right)\left(\gamma_{A}+\mu \right)}{\alpha \sigma \left(\gamma_{A}+\mu \right)+\left(1-\alpha \right)\eta \sigma \left(\sigma +\tau +\mu \right)}. \end{array}$$

We alter the initial design of the state model (1) for easy computations as follows; *S* = *x*_1_, *E* = *x*_2_, *Q* = *x*_3_, *I* = *x*_4_, *A* = *x*_5_, *H* = *x*_6_, and *R* = *x*_7_, such that *N* = *x*_1_ + *x*_2_ + *x*_4_ + *x*_5_ + *x*_7_. Also, *X* = (*x*_1_, *x*_2_, ⋯,*x*_7_)^*T*^ and *f* = (*f*_1_, *f*_2_, ⋯,*f*_7_)^*T*^ are vector notations of the model system (1) and can be rewritten in the form

(31) $$\begin{array}{c} \frac{d}{dt}x=f\left(x,\beta^{*}\right), \end{array}$$

where

(32) $$\begin{array}{c} \overset{7}{\underset{i=1}{\sum }}f_{i}=\frac{d}{dt}x_{i}=\left\{\begin{array}{c} \frac{d}{dt}x_{1}=\Lambda -\frac{\beta x_{1}x_{4}}{\sum_{i=1}^{n}\;x_{i}}-\frac{\beta x_{1}\eta x_{5}}{\sum_{i=1}^{n}\;x_{i}}-\mu x_{1},\\ \frac{d}{dt}x_{2}=\frac{\beta x_{1}x_{4}}{\sum_{i=1}^{n}\;x_{i}}+\frac{\beta x_{1}\eta x_{5}}{\sum_{i=1}^{n}\;x_{i}}-\sigma E-\tau x_{2}-\mu x_{2},\\ \frac{d}{dt}x_{3}=\tau x_{2}-\left(\tau_{1}+\mu \right)x_{3},\\ \frac{d}{dt}x_{4}=\alpha \sigma x_{2}-\phi x_{4}-\gamma_{I}x_{4}-\mu x_{4},\\ \frac{d}{dt}x_{5}=\left(1-\alpha \right)\sigma x_{2}-\gamma_{A}x_{5}-\mu x_{5},\\ \frac{d}{dt}x_{6}=\tau_{1}x_{3}+\phi x_{4}-\delta x_{6}-\gamma_{H}x_{6}-\mu x_{6},\\ \frac{d}{dt}x_{7}=\gamma_{I}x_{4}+\gamma_{A}x_{5}+\gamma_{H}x_{6}-\mu x_{7}. \end{array}\right. \end{array}$$

Now, the Jacobian matrix of model system (1) was evaluated at *E*_0_, when *β* = *β*^∗^ is provided as

(33) $$\begin{array}{c} {\left.J_{E_{0}}\right|}_{\beta =\beta^{*}}=\left[\begin{array}{ccccccc} -\mu & 0 & 0 & -\beta^{*} & -\beta^{*}\eta & 0 & 0\\ 0 & -\left(\sigma +\mu \right) & 0 & -\beta^{*} & -\beta^{*}\eta & 0 & 0\\ 0 & -\tau & -\left(\tau_{1}+\mu \right) & 0 & 0 & 0 & 0\\ 0 & \alpha \sigma & 0 & -\left(\phi +\gamma_{I}+\mu \right) & 0 & 0 & 0\\ 0 & \left(1-\alpha \right)\sigma & 0 & 0 & -\left(\gamma_{A}+\mu \right) & 0 & 0\\ 0 & 0 & \tau_{1} & \phi & 0 & -\left(\delta +\gamma_{H}+\mu \right) & 0\\ 0 & 0 & 0 & \gamma_{I} & \gamma_{A} & \gamma_{H} & -\mu \end{array}\right]. \end{array}$$

The Jacobian matrix *J*_*E*_0__|_*β*=*β*^∗^_ has a right eigenvector corressponding to a simple zero eigenvalue given by *𝒲* = (*w*_1_, *w*_2_, ⋯,*w*_7_)^*T*^ and a left eigenvector corressponding to a simple eigenvalue given by *𝒱* = (*v*_1_, *v*_2_, ⋯,*v*_7_)^*T*^. Deducing the eigenvectors of *𝒲* and *𝒱* gives

(34) $$\begin{array}{c} w_{1}=-\frac{\alpha \sigma \beta^{*}w_{2}}{\mu \left(\phi +\gamma_{I}+\mu \right)}-\frac{\left(1-\alpha \right)\sigma \beta^{*}w_{2}}{\left(\gamma_{A}+\mu \right)}, \end{array}$$

(35) $$\begin{array}{c} v_{1}=v_{7}=0,v_{2}>0,v_{3}=0,v_{6}=0,v_{4}=\frac{\beta^{*}v_{2}}{\left(\phi +\gamma_{I}+\mu \right)},v_{5}=\frac{\beta^{*}v_{2}}{\left(\gamma_{A}+\mu \right)}. \end{array}$$

The derivation of the nonzero partial derivatives is given by

(36) $$\begin{array}{c} \frac{\partial^{2}f_{2}}{\partial x_{1}\partial x_{4}}=-\alpha v_{2}{\left(\beta^{*}\right)}^{2}\sigma^{2}{w_{2}}^{2}\left(\frac{\alpha \left(\gamma_{A}+\mu \right)+\left(1-\alpha \right)\left(\phi +\gamma_{I}+\mu \right)\mu }{\mu {\left(\phi +\gamma_{I}+\mu \right)}^{2}\left(\gamma_{A}+\mu \right)}\right),\\ \frac{\partial^{2}f_{2}}{\partial x_{1}\partial x_{5}}=-v_{2}{\left(\beta^{*}\right)}^{2}\eta \sigma^{2}{w_{2}}^{2}\left(1-\alpha \right)\left(\frac{\alpha \left(\gamma_{A}+\mu \right)+\left(1-\alpha \right)\left(\phi +\gamma_{I}+\mu \right)\mu }{\mu {\left(\phi +\gamma_{I}+\mu \right)}^{2}\left(\gamma_{A}+\mu \right)}\right),\\ \frac{\partial^{2}f_{2}}{\partial x_{4}\partial \beta^{*}}=\left(\frac{v_{2}\alpha \sigma \Lambda w_{2}}{\mu \left(\phi +\gamma_{I}+\mu \right)}\right),\\ \frac{\partial^{2}f_{2}}{\partial x_{5}\partial \beta^{*}}=\frac{\Lambda v_{2}\left(1-\alpha \right)\sigma w_{2}}{\mu \left(\gamma_{A}+\mu \right)}. \end{array}$$

Hence, we obtain

(37) $$\begin{array}{c} a=-v_{2}{\left(\beta^{*}\right)}^{2}\eta \sigma^{2}{w_{2}}^{2}\left(1-\alpha \right)\left(\alpha \left(\gamma_{A}+\mu \right)+\left(1-\alpha \right)\left(\phi +\gamma_{I}+\mu \right)\mu \right)\left(\frac{\alpha \left(\gamma_{A}+\mu \right)+\left(1-\alpha \right)\left(\phi +\gamma_{I}+\mu \right)\mu }{\mu {\left(\phi +\gamma_{I}+\mu \right)}^{2}\left(\gamma_{A}+\mu \right)}\right),\\ b=v_{2}\sigma \Lambda w_{2}\left(\frac{\alpha \left(\gamma_{A}+\mu \right)+\left(1-\alpha \right)\left(\phi +\gamma_{I}+\mu \right)\mu }{\mu \left(\phi +\gamma_{I}+\mu \right)\left(\gamma_{A}+\mu \right)}\right). \end{array}$$

The coefficient *b* is positive as always. According to Theorem 6 of Castillo-Chavez and Song [69], the sign of *a* determines the local dynamics around the disease-free equilibrium for *β* = *β*^∗^.

## 4. COVID-19 Optimal Control Model

In formulating the optimal control model, we restructure the compartmental model (1) into an optimal control model with admissible controls that are considered to be continuous in time. The controls that are identified for the new structured control model are defined as follows:

*F1*. The personal protection control rate varies with time and is given by *n*_1_.

*F2*. The vaccination control rate varies with time and is denoted as *n*_2_.

*F3*. The considered time is given by *t* ∈ [0, *T*], where *T* is the final time and relatively short.

Hence, the new restructured system for Equation (1) is provided below.

(38) $$\begin{array}{c} \left\{\begin{array}{c} \frac{d}{dt}S=\Lambda -\left(1-n_{1}\right)\frac{\beta SI}{N}-\left(1-n_{1}\right)\frac{\beta S\eta A}{N}-\mu S-n_{2}S,\\ \frac{d}{dt}E=\left(1-n_{1}\right)\frac{\beta SI}{N}+\left(1-n_{1}\right)\frac{\beta S\eta A}{N}-\sigma E-\tau E-\mu E,\\ \frac{d}{dt}Q=\tau E-\left(\tau_{1}+\mu \right)Q,\\ \frac{d}{dt}I=\alpha \sigma E-\phi I-\gamma_{I}I-\mu I,\\ \frac{d}{dt}A=\left(1-\alpha \right)\sigma E-\gamma_{A}A-\mu A,\\ \frac{d}{dt}H=\phi I+\tau_{1}Q-\delta H-\gamma_{H}H-\mu H,\\ \frac{d}{dt}R=\gamma_{I}I+\gamma_{A}A+\gamma_{H}H+n_{2}S-\mu R, \end{array}\right. \end{array}$$

with *S* ≥ 0, *E* ≥ 0, *Q* ≥ 0, *I* ≥ 0, *A* ≥ 0, *H* ≥ 0, and *R* ≥ 0.

We usher in a measurable control set:

(39) $$\begin{array}{c} C≔\left\{n=\left(n_{1},n_{2}\right)\left|n_{j}\right.\left(t\right)\text{ is Lebesgue measurable},0\leq n_{i}\left(t\right)\leq 1,t\in \left[0,t_{f}\right]\text{ for }j=1,2.\right\}. \end{array}$$

The target of the considered control strategy is to

- Lower the COVID exposed, asymptomatic, and symptomatic infectious persons
- Make intervention cost small as possible

In achieving the intended goals, we design an objective functional below as in ([57, 71]).

(40) $$\begin{array}{c} J=\int_{0}^{t_{f}}\left[\nu_{1}E+\nu_{2}I+\nu_{3}A+\frac{1}{2}h_{1}n_{1}^{2}+\frac{1}{2}h_{2}n_{2}^{2}\right].dt. \end{array}$$

The constants *ν*_1_, *ν*_2_, and *ν*_3_ are weight related to exposed, symptomatic infectious, and asymptomatic infectious individuals, respectively. Additionally, the weights *h*_1_ and *h*_2_ are positive and in association with time-dependent control functions *n*_1_, *n*_2_, respectively.

The main objective of the control mode is to identify an optimal control pair *n*^∗^ = (*n*_1_^∗^, *n*_2_^∗^) that makes

(41) $$\begin{array}{c} J\left(n^{*}\right)=\underset{N}{\min}J\left(n_{1},n_{2}\right). \end{array}$$

The fundamental concept of the optimal control problem requires that we verify the existence and uniqueness of the optimal controls to characterize them.

### 4.1. Existence of Optimal Controls

As noted in [72], the existence result of Fleming and Richel is considered to show the existence of optimal control duple that minimizes (40) subject to the system (38).

**Theorem 5 .**

An optimal control duple (*n*^∗^) exists that minimizes the objective functional (40) subject to the system (38), given that the below properties are met.

- The set of control is convex and closed
- The system (38) is bounded by a linear function in both the state and control variable
- The objective functional (40) integrand is convex with respect to the control
- There exist constants *b*_1_, *b*_2_ ≥ 0, and *b*_3_ ≥ 1 that make the objective functional (40) integrand bounded by the below quantity

(42) $$\begin{array}{c} b_{1}{\left(\overset{2}{\underset{i=1}{\sum }}{\left|n_{i}\right|}^{2}\right)}^{b_{3}/2}-b_{2}. \end{array}$$

**Proof**

- It is sufficient to write *n* = *n*_1_ × *n*_2_ by definition of (39). Hence, *n* = *n*_1_ × *n*_2_ is bounded and convex ∀*t* ∈ [0, *T*]. In addition, we choose *k*, *d* ∈ *N*, so that *k* = (*k*_1_, *k*_2_) and *d* = (*d*_1_, *d*_2_). Then, ∀*v* ∈ [0, 1], and we have *vk*_*i*_ + (1 − *v*)*d*_*i*_ ∈ *N*, satisfying the convexity property of the control set
- We denote the right side of system (38) and the associated solution by *f* and *θ*; then,

(43) $$\begin{array}{c} \psi =\begin{array}{c} \left|\left[\begin{array}{c} -\left(1-n_{1}\right)\beta \left(\frac{S_{1}I_{1}}{N}-\frac{S_{2}I_{2}}{N}\right)-\left(1-n_{1}\right)\beta \eta \left(\frac{S_{1}A_{1}}{N}-\frac{S_{2}A_{2}}{N}\right)\\ -\mu \left(S_{1}-S_{2}\right)-n_{2}\left(S_{1}-S_{2}\right)\\ \left(1-n_{1}\right)\beta \left(\frac{S_{1}I_{1}}{N}-\frac{S_{2}I_{2}}{N}\right)+\left(1-n_{1}\right)\beta \eta \left(\frac{S_{1}A_{1}}{N}-\frac{S_{2}A_{2}}{N}\right)\\ -\sigma \left(E_{1}-E_{2}\right)-\tau \left(E_{1}-E_{2}\right)\\ -\mu \left(E_{1}-E_{2}\right)\\ \tau \left(E_{1}-E_{2}\right)-\left(\tau_{1}+\mu \right)\left(Q_{1}-Q_{2}\right)\\ \alpha \sigma \left(E_{1}-E_{2}\right)-\phi \left(I_{1}-I_{2}\right)-\gamma_{I}\left(I_{1}-I_{2}\right)-\mu \left(I_{1}-I_{2}\right)\\ \left(1-\alpha \right)\sigma \left(E_{1}-E_{2}\right)-\gamma_{A}\left(A_{1}-A_{2}\right)-\mu \left(A_{1}-A_{2}\right)\\ \phi \left(I_{1}-I_{2}\right)+\tau_{1}\left(Q_{1}-Q_{2}\right)-\delta \left(H_{1}-H_{2}\right)-\gamma_{H}\left(H_{1}-H_{2}\right)\\ -\mu \left(H_{1}-H_{2}\right)\\ \gamma_{I}\left(I_{1}-I_{2}\right)+\gamma_{A}\left(A_{1}-A_{2}\right)+n_{2}\left(S_{1}-S_{2}\right)-\mu \left(R_{1}-R_{2}\right) \end{array}\right]\right|, \end{array} \end{array}$$

where *ψ* = |*f*(*t*, *θ*_1_, *n*) − *f*(*t*, *θ*_2_, *n*)|

(44) $$\begin{array}{c} \leq 2\beta \left(1-n_{1}\right)\left|\left(\frac{S_{1}I_{1}}{N}-\frac{S_{2}I_{2}}{N}\right)\right|+2\beta \eta \left(1-n_{1}\right)\left|\left(\frac{S_{1}A_{1}}{N}-\frac{S_{2}A_{2}}{N}\right)\right|+2\tau \left|E_{1}-E_{2}\right|+2\sigma \left|E_{1}-E_{2}\right|+2\alpha \sigma \left|E_{1}-E_{2}\right|+2\tau_{1}\left|Q_{1}-Q_{2}\right|+2\gamma_{A}\left|A_{1}-A_{2}\right|+2\gamma_{H}\left|H_{1}-H_{2}\right|+2n_{2}\left|S_{1}-S_{2}\right|+2\phi \left|I_{1}-I_{2}\right|+\mu \left|S_{2}-S_{1}\right|+\mu \left|E_{2}-E_{1}\right|+\mu \left|Q_{2}-Q_{1}\right|+\mu \left|I_{2}-I_{1}\right|+\mu \left|A_{2}-A_{1}\right|+\mu \left|H_{2}-H_{1}\right|+\mu \left|R_{2}-R_{1}\right|,\\ \leq 2\beta \left(1-n_{1}\right)\left|I_{1}\left(S_{1}-S_{2}\right)+S_{2}\left(I_{1}-I_{2}\right)\right|+2\beta \eta \left(1-n_{1}\right)\left|A_{1}\left(S_{1}-S_{2}\right)+S_{2}\left(A_{1}-A_{2}\right)\right|+\left(2\tau +2\sigma +2\alpha +2\alpha \sigma +\mu \right)\left|E_{1}-E_{2}\right|+\left(2\tau_{1}+\mu \right)\left|Q_{1}-Q_{2}\right|+\left(2\gamma_{A}+\mu \right)\left|A_{1}-A_{2}\right|+\left(2\gamma_{H}+\mu \right)\left|H_{1}-H_{2}\right|+\left(2n_{2}+\mu \right)\left|S_{1}-S_{2}\right|+\left(2\phi +\mu \right)\left|I_{1}-I_{2}\right|+\mu \left|R_{2}-R_{1}\right|,\\ \leq \left|S_{1}-S_{2}\right|\left(2\beta \left(1-n_{1}\right)\left|I_{1}\right|+2\beta \eta \left(1-n_{1}\right)\left|A_{1}\right|\right)+2\beta \left(1-n_{1}\right)\left|S_{2}\right|\left|I_{1}-I_{2}\right|+2\beta \eta \left(1-n_{1}\right)\left|S_{2}\right|\left|A_{1}-A_{2}\right|+\left(2\tau +2\sigma +2\alpha +2\alpha \sigma +\mu \right)\left|E_{1}-E_{2}\right|+\left(2\tau_{1}+\mu \right)\left|Q_{1}-Q_{2}\right|+\left(2\gamma_{A}+\mu \right)\left|A_{1}-A_{2}\right|+\left(2\gamma_{H}+\mu \right)\left|H_{1}-H_{2}\right|+\left(2n_{2}+\mu \right)\left|S_{1}-S_{2}\right|+\left(2\phi +\mu \right)\left|I_{1}-I_{2}\right|+\mu \left|R_{2}-R_{1}\right|,\\ \leq \left(2n_{2}+\mu \right)\left|S_{1}-S_{2}\right|+\left(2\tau +2\sigma +2\alpha +2\alpha \sigma +\mu \right)\left|E_{1}-E_{2}\right|+\left(2\tau_{1}+\mu \right)\left|Q_{1}-Q_{2}\right|+\left(2\beta \frac{\Lambda }{\mu }\left(1-n_{1}\right)+2\phi +\mu \right)\left|I_{1}-I_{2}\right|+\left(2\beta \frac{\eta \Lambda }{\mu }\left(1-n_{1}\right)+2\gamma_{A}+\mu \right)\left|A_{1}-A_{2}\right|+\left(2\gamma_{H}+\mu \right)\left|H_{1}-H_{2}\right|+\mu \left|R_{2}-R_{1}\right|,\\ \leq G_{1}\left|S_{1}-S_{2}\right|+G_{2}\left|E_{1}-E_{2}\right|+G_{3}\left|Q_{1}-Q_{2}\right|+G_{4}\left|I_{1}-I_{2}\right|+G_{5}\left|A_{1}-A_{2}\right|+G_{6}\left|H_{1}-H_{2}\right|+G_{7}\left|R_{1}-R_{2}\right|, \end{array}$$

where *G*_1_ = (2*n*_2_ + *μ*), *G*_2_ = (2*τ* + 2*σ* + 2*ασ* + *μ*), *G*_3_ = (2*τ*_1_ + *μ*), *G*_4_ = (2(*βΛ*/*μ*)(1 − *n*_1_) + 2*ϕ* + *μ*), *G*_5_ = (2(*βηΛ*/*μ*)(1 − *n*_1_) + 2*γ*_*A*_ + *μ*), *G*_6_ = (2*γ*_*A*_ + *μ*), *G*_7_ = *μ*, and *G* = max{*G*_1_, *G*_2_, *G*_3_, *G*_4_, *G*_5_, *G*_6_, *G*_7_}.

Hence, *f* is uniformly Lipschitz continuous.

(c) The Langrangian defined as *L*(*t*, *z*, *n*) is the integrand of the objective functional (40). Thus, we rewrite *L*(*t*, *z*, *n*) in the form

(45) $$\begin{array}{c} L\left(t,z,n\right)=r_{1}\left(t,z\right)+r_{2}\left(t,z\right), \end{array}$$

with

*r*_1_(*t*, *z*) = *ν*_1_*E* + *ν*_2_*I* + *ν*_3_*A* and *r*_2_(*t*, *z*) = 1/2∑_*j*=1_^2^*h*_*j*_*n*_*j*_. The convexity of *r*_2_(*t*, *z*), which is a linear combination of the control function 1/2∑_*j*=1_^2^*h*_*j*_*n*_*j*_, needs to be proved. We prove the convexity by letting *c* : [0, 1]^2^⟶*R* be *h*(*n*) = 1/2*n*^2^. Then, ∀*u*_1_, *u*_2_ ∈ [0, 1]^2^ and *ρ* ∈ [0, 1]. Hence, it follows that the below inequality holds.

(46) $$\begin{array}{c} \rho c\left(u_{1}\right)+\left(1-\rho \right)c\left(u_{2}\right)\geq c\left(\rho u_{1}+\left(1-\rho \right)u_{2}\right). \end{array}$$

This confirms the convexity of the Langrangian with respect to the control.

(d) When observed from (45), we easily see that *L*(*t*, *z*, *n*) ≥ *r*_1_(*t*, *z*). Hence, we conclude that

(47) $$\begin{array}{c} L\left(t,z,n\right)\geq \frac{1}{2}h_{1}n_{1}^{2}+\frac{1}{2}h_{2}n_{2}^{2}\geq b_{1}{\left(\overset{2}{\underset{i=1}{\sum }}{\left|n_{i}\right|}^{2}\right)}^{b_{3}/2}-b_{2}, \end{array}$$

with *b*_1_ = 1/2min{*h*_1_, *h*_2_}, *b*_2_ > 0, and *b*_3_ = 2. This completes the proof.

### 4.2. Characterization of Optimal Controls

Pontryagin's maximum principle has been the wheel on which the necessary condition for the COVID (38) duple control needs to meet. With the principle, we convert the COVID (38) and the objective functional (40) into a problem of minimizing the Hamiltonian *H*_*f*_ with respect to the controls *n*_*j*_(*t*), *j* = 1, 2. Hence, the Hamiltonian *H*_*f*_ is given by

(48) $$\begin{array}{c} H_{f}=\left[\nu_{1}E+\nu_{2}I+\nu_{3}A+\frac{1}{2}h_{1}n_{1}^{2}+\frac{1}{2}h_{2}n_{2}^{2}\right]+\zeta_{1}\left\{\Lambda -\left(1-n_{1}\right)\frac{\beta SI}{N}-\left(1-n_{1}\right)\frac{\beta S\eta A}{N}-\mu S-n_{2}S\right\}+\zeta_{2}\left\{\left(1-n_{1}\right)\frac{\beta SI}{N}+\left(1-n_{1}\right)\frac{\beta S\eta A}{N}-\sigma E-\tau E-\mu E\right\}+\zeta_{3}\left\{\tau E-\left(\tau_{1}+\mu \right)Q\right\}+\zeta_{4}\left\{\alpha \sigma E-\phi I-\gamma_{I}I-\mu I\right\}+\zeta_{5}\left\{\left(1-\alpha \right)\sigma E-\gamma_{A}A-\mu A\right\}+\zeta_{6}\left\{\phi I+\tau_{1}Q-\delta H-\gamma_{H}H-\mu H\right\}+\zeta_{7}\left\{\gamma_{I}I+\gamma_{A}A+\gamma_{H}H+n_{2}S-\mu R\right\}. \end{array}$$

**Theorem 6 .**

With the optimal control duple (*n*_1_^∗^, *n*_2_^∗^) satisfying the condition (41), there exist adjoint variables *ζ*_*i*_ satisfying the adjoint system below.

(49) $$\begin{array}{c} \frac{d\zeta_{1}}{dt}=\left(\zeta_{1}-\zeta_{2}\right)\left(1-n_{1}\right)\beta I\frac{\left(\left(S+E+I+A+R\right)+S\right)}{N^{2}}+\left(\zeta_{1}-\zeta_{2}\right)\left(1-n_{1}\right)\beta \eta A\frac{\left(\left(S+E+I+A+R\right)+S\right)}{N^{2}}+\left(\zeta_{1}-\zeta_{7}\right)n_{2}+\mu \zeta_{1},\\ \frac{d\zeta_{2}}{dt}=-\nu_{1}+\left(\zeta_{2}-\zeta_{1}\right)\frac{\beta SI}{N^{2}}+\left(\zeta_{2}-\zeta_{1}\right)\left(1-n_{1}\right)\frac{\beta \eta SA}{N^{2}}+\left(\zeta_{2}-\zeta_{5}\right)\sigma +\left(\zeta_{2}-\zeta_{3}\right)\tau +\left(\zeta_{5}-\zeta_{4}\right)\alpha \sigma +\mu \zeta_{2},\\ \frac{d\zeta_{3}}{dt}=\left(\zeta_{3}-\zeta_{6}\right)\tau_{1}+\mu \zeta_{3},\\ \frac{d\zeta_{4}}{dt}=-\nu_{2}+\left(\zeta_{1}-\zeta_{2}\right)\left(1-n_{1}\right)\beta S\frac{\left(\left(S+E+I+A+R\right)+I\right)}{N^{2}}+\left(\zeta_{2}-\zeta_{1}\right)\left(1-n_{1}\right)\frac{\beta \eta SA}{N^{2}}+\left(\zeta_{4}-\zeta_{6}\right)\phi +\left(\zeta_{4}-\zeta_{7}\right)\gamma_{I}+\mu \zeta_{4},\\ \frac{d\zeta_{5}}{dt}=-\nu_{3}+\left(\zeta_{1}-\zeta_{2}\right)\left(1-n_{1}\right)\beta \eta A\frac{\left(\left(S+E+I+A+R\right)+A\right)}{N^{2}}+\frac{\left(\zeta_{2}-\zeta_{1}\right)\beta SI}{N^{2}}+\left(\zeta_{5}-\zeta_{7}\right)\gamma_{A}+\mu \zeta_{5},\\ \frac{d\zeta_{6}}{dt}=\left(\zeta_{6}-\zeta_{7}\right)\gamma_{H}+\delta \zeta_{6}+\mu \zeta_{6},\\ \frac{d\zeta_{7}}{dt}=\left(\zeta_{2}-\zeta_{1}\right)\frac{\beta SI}{N^{2}}+\left(\zeta_{2}-\zeta_{1}\right)\frac{\beta \eta SA}{N^{2}}+\mu \zeta_{7}, \end{array}$$

with transversality conditions

(50) $$\begin{array}{c} \zeta_{j}\left(T\right)=0,j\in \left\{1,2,3,4,5,6,7\right\}, \end{array}$$

with control functions (*n*_1_^∗^, *n*_2_^∗^) which satisfy the optimality condition given by

(51) $$\begin{array}{c} \left\{\begin{array}{c} n_{1}^{\prime }\left(t\right)=\min\left\{1,\max\left\{0,\left(\left(\zeta_{2}-\zeta_{1}\right)\frac{\beta \left(I+\eta A\right)S}{h_{1}N}\right)\right\}\right\},\\ n_{2}^{\prime }\left(t\right)=\min\left\{1,\max\left\{0,\left(\left(\zeta_{1}-\zeta_{7}\right)\frac{S}{h_{2}}\right)\right\}\right\}. \end{array}\right. \end{array}$$

**Proof**

With reference to the Hamiltonian (48), the adjoint system (49) is determined by partially differentiating the Hamiltonian (48) with respect to the corresponding state variables *S*, *E*, *Q*, *I*, *A*, *H*, *R* as

(52) $$\begin{array}{c} \frac{d\zeta_{1}}{dt}=-\frac{\partial H_{f}}{\partial S},\\ \frac{d\zeta_{2}}{dt}=-\frac{\partial H_{f}}{\partial E},\\ \frac{d\zeta_{3}}{dt}=-\frac{\partial H_{f}}{\partial Q},\\ \frac{d\zeta_{4}}{dt}=-\frac{\partial H_{f}}{\partial I},\\ \frac{d\zeta_{5}}{dt}=-\frac{\partial H_{f}}{\partial A},\\ \frac{d\zeta_{6}}{dt}=-\frac{\partial H_{f}}{\partial H},\\ \frac{d\zeta_{7}}{dt}=-\frac{\partial H_{f}}{\partial R}. \end{array}$$

The characterization of the controls of (51) are derived by solving *n*_1_^∗^ and *n*_2_^∗^ from the equation below.

(53) $$\begin{array}{c} \left\{\begin{array}{c} \frac{\partial H_{f}}{\partial n_{1}}=0,\\ \frac{\partial H_{f}}{\partial n_{2}}=0. \end{array}\right. \end{array}$$

Applying bounds on the controls by standard argument, we deduce the characterization.

(54) $$\begin{array}{c} n_{i}^{*}=\left\{\begin{array}{cc} 0 & \text{if }\omega_{i}^{*}\leq 0,\\ w_{i}^{*} & \text{if }0\leq \omega_{i}^{*}\leq 1,\\ 1 & \text{if }\omega_{i}^{*}\geq 1, \end{array}\right. \end{array}$$

where

(55) $$\begin{array}{c} \omega_{1}^{*}=\left(\left(\zeta_{2}-\zeta_{1}\right)\frac{\beta \left(I+\eta A\right)S}{h_{1}N}\right),\\ \omega_{2}^{*}=\left(\left(\zeta_{1}-\zeta_{7}\right)\frac{S}{h_{2}}\right). \end{array}$$

Hence. the proof is complete.

## 5. Model Application with Numerical Examples

As credited to Lenhart and Workman [73], the method of forward-backward sweep has been explored extensively by many researchers as in [74–76] to solve the optimality system of optimal control models numerically. Hence, we consider the method to solve the COVID-19 (1) and the control system (38). We design numerical scheme that uses Runge-Kutta's fourth-order method [70, 77, 78] to solve the model's optimality system. The optimality system results and the control problem's state system are numerically obtained by the Runge-Kutta method of order four, with Matlab. The constants *ν*_1_ = 10, *ν*_2_ = 8, *ν*_3_ = 5, *h*_1_ = 5, and *h*_2_ = 10 were used to balance the terms of the objective functional's equation, and we utilized the parameter values presented in Table 1 to generate the plots of symptomatic infectious, exposed, and asymptomatic infectious. The weight *h*_2_ > *h*_1_, since we assume that the cost of vaccinating the population would be greater than the self-protection strategy.

### 5.1. Strategy A (with *n*_1_ and *n*_2_)

In an effort to curtail the pandemic, the controls *n*_1_ and *n*_2_ were utilized. The plots of the graphs of Figures 1(a)–1(c) showed an increase in the number of exposed, symptomatic, and asymptomatic infectious individuals in the first 20, 30, and 30 days, respectively, for the noncontrol case. The noncontrol exposed curve rises sharply in the first 5 days until about the 20 days, where its dynamic changes gradually decrease. In a like manner, the symptomatic and asymptomatic infectious curves quickly rise in the early days until 40 days when their dynamics change and begin to decrease. Notwithstanding, utilizing the controls *n*_1_ and *n*_2_, we notice that the number of exposed, symptomatic, and asymptomatic infectious individuals is greatly minimized. Furthermore, the exposed, symptomatic graphs drop gradually for the first 20 until they completely wipe out the population in 80 and 120 days, respectively. This shows the optimal control strategy's effectiveness as it has a substantial effect of drastically minimizing the exposed, symptomatic, and asymptomatic graphs.  Figure 1(d) depicts the strategy A's control profile. We noticed that the personal protection control *n*_1_ and vaccination control *n*_2_ stayed at the upper bound throughout the simulated time of 180 days.

### 5.2. Strategy B (with *n*_1_)

Owing to the effort to curtail the disease from spreading, we utilized controls *n*_1_. The plot of the graphs of Figures 2(a)–2(c) of the noncontrol model indicated an increase in the number of exposed, symptomatic, and asymptomatic infectious individuals in the first 10, 35, and 30 days of the simulated time. The exposed graph of (a) quickly rises in the first 10 days until it reaches a maximum height of about 800 when it suddenly changes its dynamics and begins to decrease. The symptomatic and asymptomatic infectious graphs similarly rise in the early days of the simulated time and drop after 35 days. However, with the optimal control strategy of *n*_1_, the desired result of minimizing the exposed, symptomatic, and asymptomatic infectious individuals is obtained. Thus, in a similar pattern, even though the control graphs rose early and reached the height of the noncontrol plots, they were lowered than the noncontrol graphs in the final run. This means that the strategy of the controls *n*_1_ is efficient for preventing the further spread of the disease, even though it does not bring out the best result. In Figure 2(d), we have a clear view of strategy B's control profile. As noticed, the control profile of the personal protection control *n*_1_ stayed at the middle throughout the simulated time of 180 days.

### 5.3. Strategy C (with *n*_2_)

We considered the control *n*_2_ in an attempt to defeat the pandemic. The simulated plot of the noncontrol graphs of Figures 3(a)–3(c) indicated an early increase in the number of the exposed, symptomatic, and asymptomatic individuals at the estimated time of about 20, 30, and 30 days, respectively. The situation is reversed with the application of an optimal control strategy. With *n*_2_, the plots produced results of the exposed, symptomatic, and asymptomatic individuals' graphs greatly minimized. Even though the asymptomatic individual's optimal control plot rises quickly, similar to the noncontrol plot, the control strategy is considered efficient as it minimizes the asymptomatic infectious individuals substantially.  Figure 3(d) shows the strategy C's control profile. We observed that the vaccination control *n*_1_ was at the upper bound throughout the simulated time of 180 days.

### 5.4. Conclusion

This research article presented a SEQIAHR compartmental model of COVID-19 to provide insight into the disease's dynamics by utilizing tailored strategies to minimize the pandemic. We first studied the COVID nonlinear model's dynamic behaviour by calculating the reproduction number and examining the two nonnegative equilibria's existence. Global stability analyses for the two equilibria were also carried out by employing the Castillo-Chavez method and Lyapunov function to investigate the global stability of the disease at the disease-free and endemic equilibrium. We carried out a sensitivity analysis on the model to determine the parameters that have relative effects on the *R*_0_. We examined the model system (1) to determine the type of bifurcation that it exhibits. Then, we formulated a new SEQIAHR compartmental optimal control model with time-dependent controls: personal protection and vaccination of susceptible individuals and solved it utilizing Pontryagin's maximum principle after studying the dynamical behaviour of the noncontrol model. We solved the model numerically by considering different simulation controls' pairing and examined their effectiveness. The results showed that each optimal control strategy chosen has an incomparable impact on the number of the exposed, symptomatic, and asymptomatic individuals compared to the noncontrol model since they substantially minimize exposed, symptomatic, and asymptomatic infectious individuals. Thus, strategy A considered both personal protection and vaccination control. We noticed that the combined effect of the strategies had a significant impact on the disease by emphatically minimizing the exposed, symptomatic, and asymptomatic infectious individuals. Strategy B considered only the personal protection control in its intervention program. Even though, to some extent, the strategy minimized the exposed, symptomatic, and asymptomatic infectious individuals in the long run. We observed that in the early days of the graphs, the strategy struggled to minimize these individuals. In addition, the exposed, symptomatic, and asymptomatic infectious individuals are not greatly minimized. The results of strategy B mean that resorting to this intervention strategy will not bring out the desired results as individuals may refuse to adhere to the personal protection protocols as directed by stakeholders and may put the entire population at risk of the pandemic. Strategy C employed the vaccination control as the only control for its intervention program. However, we obtained a great result as the exposed, symptomatic, and asymptomatic infectious individuals are substantially minimized. The result showed that using only vaccination as the control intervention could have the same mitigating effect on the disease as employing both personal protection and vaccination strategies with a minimized.

## Figures and Tables

**Figure 1:** Numerical solutions.

**Figure 2:** Numerical solutions.

**Figure 3:** Numerical solutions.

**Table 1:** COVID-19 model 1 equation parameters.

Parameter	Description	Value	Reference
*β*	Infection contact rate	(1.5)/day	[26]
*σ*	Transition from exposed to infectious	(1/14)/day	[26]
*η*	Infectiousness factor for asymptomatic carriers	(0.6)	[26]
*α*	Fraction of infections that become symptomatic	(0.15)	[26]
*ϕ*	Hospitalization rate	(0.02)	[26]
*γ*_*A*_	Asymptomatic (recovery rate)	(1/14)/day	[26]
*γ*_*I*_	Symptomatic (recovery rate)	(1/30)/day	[26]
*γ*_*H*_	Hospitalized (recovery rate)	(1/14)/day	[66]
*δ*	Death rate (hospitalized)	0.01	[45]
*Λ*	Recruitment rate	50	Assumed
*τ*	Quarantine rate	0.012	[60]
*τ*_1_	Hospitalized rate	0.06	[26]
*μ*	Natural death rate	0.000042578	[4]

**Table 2:** Parameters for *R*_0_ and their sensitivity index for model (1).

Parameter	Sensitivity index
*β*	+1
*σ*	-1.3094
*η*	+0.7174
*α*	+0.1560
*ϕ*	-0.1066
*γ*_*A*_	-0.0510
*γ*_*I*_	-0.1756
*τ*	-0.1445
*μ*	-0.00010

## Data Availability

The authors declare that our mathematical modelling does not include data. All parameter values that were used for our simulations have been cited accordingly.
